# High prevalence of carriers of variant c.1528G>C of *HADHA* gene causing long-chain 3-hydroxyacyl-CoA dehydrogenase deficiency (LCHADD) in the population of adult Kashubians from North Poland

**DOI:** 10.1371/journal.pone.0187365

**Published:** 2017-11-02

**Authors:** Bogusław Nedoszytko, Alicja Siemińska, Dominik Strapagiel, Sławomir Dąbrowski, Marcin Słomka, Marta Sobalska-Kwapis, Błażej Marciniak, Jolanta Wierzba, Jarosław Skokowski, Marcin Fijałkowski, Roman Nowicki, Leszek Kalinowski

**Affiliations:** 1 Department of Dermatology, Venereology and Allergology, Medical University of Gdansk, Gdańsk, Poland; 2 Department of Pneumonology and Allergology, Medical University of Gdansk, Gdańsk, Poland; 3 Biobank Lab, Department of Molecular Biophysics, Faculty of Biology and Environmental Protection, University of Lodz, Lodz, Poland; 4 BBMRI.pl Consortium, Wrocław, Poland; 5 A&A Biotechnology s.c., Gdynia, Poland; 6 Department of Pediatrics, Hematology and Oncology, Medical University of Gdansk, Gdańsk, Poland; 7 Department of Oncological Surgery, Medical University of Gdansk, Gdańsk, Poland; 8 I Department of Cardiology, Medical University of Gdansk, Gdańsk, Poland; 9 Department of Medical Laboratory Diagnostic, Central Bank of Frozen Tissues and Genetic Specimens, Medical University of Gdansk, Gdańsk, Poland; University of Alabama at Birmingham, UNITED STATES

## Abstract

**Background/Objectives:**

The mitochondrial β-oxidation of fatty acids is a complex catabolic pathway. One of the enzymes of this pathway is the heterooctameric mitochondrial trifunctional protein (MTP), composed of four α- and β-subunits. Mutations in MTP genes (*HADHA* and *HADHB*), both located on chromosome 2p23, cause MTP deficiency, a rare autosomal recessive metabolic disorder characterized by decreased activity of MTP. The most common MTP mutation is long-chain 3-hydroxyacyl-CoA dehydrogenase (LCHAD) deficiency caused by the c.1528G>C (rs137852769, p.Glu510Gln) substitution in exon 15 of the *HADHA* gene.

**Subjects/Methods:**

We analyzed the frequency of genetic variants in the *HADHA* gene in the adults of Kashubian origin from North Poland and compared this data in other Polish provinces.

**Results:**

We found a significantly higher frequency of HDHA c.1528G>C (rs137852769, p.Glu510Gln) carriers among Kashubians (1/57) compared to subjects from other regions of Poland (1/187). We found higher frequency of c.652G>C (rs71441018, pVal218Leu) polymorphism in the HADHA gene within population of Silesia, southern Poland (1/107) compared to other regions.

**Conclusion:**

Our study indicate described high frequency of c.1528G>C variant of *HADHA* gene in Kashubian population, suggesting the founder effect. For the first time we have found high frequency of rs71441018 in the South Poland Silesian population.

## Introduction

The mitochondrial β-oxidation of fatty acids is a complex catabolic pathway in which at least 10 different enzymes are involved. One of the last enzyme of this pathway is the mitochondrial trifunctional protein (MTP), a heterooctameric protein composed of four α- and four β-subunits. MTP has trifunctional enzymatic activity: it acts as long-chain enoyl-CoA hydratase (LCEH), long-chain 3-hydroxyacyl-CoA dehydrogenase (LCHAD) and long-chain 3-ketothiolase (LKCT). The LCHAD and LCEH activity is associated with its α-subunit (OMIM #600890), whereas LKCT activity is associated with the β-subunit (OMIM #143450) of MTP. The α- and β-subunits of MTP are encoded by different genes (*HADHA* and *HADHB*), both located on chromosome 2p23 [1]. The most common MTP deficiency in Europe is the isolated long-chain 3-hydroxyacyl-CoA dehydrogenase (LCHAD) deficiency caused by c.1528G>C substitution on at least one allele of the *HADHA* gene [1–12].

Isolated long-chain 3-hydroxyacyl-CoA dehydrogenase deficiency (LCHADD, OMIM#609016) is an autosomal recessive disorders associated with mutations of the *HADHA* gene first described in 1989 by Wanders et al.[10]. *HADHA* contains 20 exons spanning over 52 kb. More than 30 variants have been described up to date [10–12].

The most common variant in *HADHA* is a c.1528G>C substitution in exon 15, which alter glutamic acid into glutamine (p.Glu510Gln), within the catalytic region of the enzyme that causes decreased activity of the dehydrogenase activity with normal hydratase activity and moderately decreased thiolase activity [3]. This variant is observed in 87–91% of European patients with clinically overt disease. Compound heterozygosity for the c.1528G>C variant and a second *HADHA* polymorphism (for ex. p.Arg524Ter, or p.Arg255Ter) may also result in general MTP deficiency. Determination of enzymatic activity is the only way to characterize isolated LCHAD deficiency or general MTP deficiency [3, 7, 8, 13].

Isolated LCHAD deficiency in children may be associated with severe maternal illness occurring during pregnancies with fetuses affected by HELLP syndrome, (Acute Fatty Liver Pregnancy (AFLP) and Hypertension, Elevated Liver Enzymes, and Low Platelet (HELLP) Syndromes) [13–15].

Most patients with LCHADD display a severe phenotype that presents itself during infancy, usually from the neonatal period until 12 months of age. The disease manifests as hypoketotic hypoglycemia, metabolic acidosis, hypotonia, liver involvement with hepatic encephalopathy, cardiomyopathy and arrhythmias, peripheral neuropathy and recurrent rhabdomyolysis. Clinical presentation is frequently preceded by fasting and/or intercurrent illness and often presents with hypoketotic hypoglycemia. Chronic peripheral neuropathy and pigmentary retinopathy develop over time in many surviving patients. Rarer presentations of LCHADD are sudden cardiac arrest or sudden infant death [3, 16].

The frequency of c.1528G>C carriers is highest in populations living near the Baltic sea, and is 1/240 in Finland, 1/680 in the Netherlands, 1/169 in Poland and 1/173 in Estonia. The birth prevalence of LCHADD is predicted to be 1/91,700 in Estonia and 1/118,336 in Poland. In comparison, the incidence was zero out of 1200 screened individuals from China and the worldwide incidence is about 1/250000-1/750000 [17–24].

Piekutowska-Abramczuk et al. found that the carriers frequency in babies born in Poland in the year 2008 was 1/217, whereas it was significantly higher in the Pomeranian region [23]. Because the majority of carriers was detected in children living in the Kashubian region, the authors suggested a probable Kashubian origin of the prevalent c.1528G>C variant. The estimated frequency of disease in the Pomeranian region was 1/16,900 whereas in rest of Poland it was 1/118,336. Kashubians are a relatively small population that inhabits Kashubia, a region in Poland’s Pomeranian Province in North Poland. Currently, the number of indigenous Kashubians is estimated at nearly 230,000. The isolation of this relatively small population is assumed to be mainly linguistic, cultural, and geographical, because its genetic structure has not been explored in detail yet. However, a high endogamy rates, slow population expansion, and insignificant immigration allows the consideration of Kashubians as a genetically isolated population [25, 26].

The aim of our study was to analyze the frequency of genetic variants in the *HADHA* gene in a sample of adult Kashubians and compare this data with the frequency found in other provinces of Poland.

## Material and methods

### Material

#### Kashubian population

The study sample was taken from the population in an isolated population of Kashubians from North Poland between October 2010 and March 2015 [26, 27]. The sample comprised of 1023 adult subjects of Kashubian origin between the age of 18 and 85 years. There were 631 (61.8%) men and 392 (38.2%) women among them. From each person 5 ml of peripheral blood were collected and stored at -70°C.

The participants were recruited from different health services from the Kashubian region of Poland (Fig 1). The Kashubian origin of participants was confirmed by being born into a Kashubian family (i.e., both mother and father, as well as four grandparents were Kashubian) and by a command of the Kashubian language.

**Fig 1:** Poland—place of origin—volunteers involved in this study.

The study protocol was approved by the Bioethics Commission of the Medical University of Gdańsk and all subjects prior to participation in the study.

#### Populations from other provinces of Poland

The participants were recruited between 2010–2012 within the TESTOPLEK research project and registered as POPULOUS collection at the Biobank Lab of The Department of Molecular Biophysics of The University of Lodz [28, 29]. Each subject gave the written informed consent and completed a questionnaire. Saliva was collected into Oragene OG-500 DNA collection/storage receptacles (DNA Genotek, Kanata, Canada) from each individual. The approval for this study was obtained from The University of Lodz’s Review Board. All procedures were performed in accordance with the Declaration of Helsinki (ethical principles for medical research involving human subjects).

From over 10,000 adult individuals throughout Poland from the POPULOUS collection, a total of 5,901 participants were involved in the creation of a study group (Fig 1). For these participants all of the survey data needed for this study was completed, including the region of saliva collection. There were 3,009 (50.99%) females and 2,892 (49.01%) males within this group, aged between 20 and 77 years (average 43.43).

### Methods

#### DNA isolation from blood samples

Genomic DNA was extracted from 100 μl of frozen blood by using the Genomic Micro AX Blood Gravity kit (A&A Biotechnology) according to the manufacturer's protocol.

#### DNA isolation from saliva samples

Genomic DNA from the participants from other regions of Poland was manually isolated from 500 μl of saliva according to the manufacturer’s protocol (PrepitL2P, PD-PR-052, DNA Genotek, Kanata, Canada). The elution volume was 50 μl. DNA was quantified using the broad range Quant-iT^™^ dsDNA Broad Range Assay Kit (Invitrogen^™^, Carlsbad, CA, USA). All DNA samples underwent quality control using a PCR reaction for sex determination [30].

#### Pyrosequencing method

The *HADHA* c.1528G>C variant was analyzed by pyrosequencing in a total of 1,023 adult subjects (Fig 2). To amplify the *HADHA* gene fragment (202 bp), primers HADHABiotFor199 (5'-[Btn]CTCACCCGCATTCTCCGAT-3') and HADHARev199 (5'-ACAGCCCCTTACCTTAACCACA-3') were used. The PCR amplification was performed using a 50 μL reaction volume containing 2 μL of genomic DNA, 2x PCR Master Mix Plus (A&A Biotechnology), and 1 μL of each primer (10 μM). The PCR used the following steps: 94°C for 3 min, followed by 40 cycles with 94°C for 15 s, 58°C for 30 s and 72°C for 30 s.; the final extension was at 72°C for 5 min. The sequencing primer was 5'-GTTTTCTCGGTCGTGATAA-3', and the nucleotide dispensation order was TCTSCAGC. Sequencing was carried out as instructed by the protocol using the PSQ^™^ 96MA pyrosequencing aparatus and the PyroMark^®^ Gold Q96 kit (Qiagen).

**Fig 2:** Pyrosequencing results indicating presence of c.1528G>C variant.

#### Microarrays analysis

The 5901 DNA samples were genotyped for 551,945 SNPs using the 24x1 Infinium HTS Human Core Exome PLUS (Illumina Inc., San Diego, CA, USA) microarrays according to the protocol provided by the manufacturer. Briefly, DNA samples were amplified, then enzymatically fragmented and hybridized to the BeadChips. Afterwards, the BeadChips underwent an extension and X-staining processes. Next the BeadChips were scanned using iScan (Illumina Inc., San Diego, CA, USA). Raw fluorescence intensities were imported to the GenomeStudio V2011.1 with the Genotyping Module v1.9.4 (Illumina Inc., San Diego, CA, USA). All data first underwent stringent quality control including sample exclusion if call rate was below 0.94 and if the 10% GenCall parameter was below 0.4. We filtered the data from the *HADHA* gene region (NC_000002.11 (26413504..26467665)) which gave 30 SNPs for the analysis. All sequence coordinates were compared to the GRCh37/hg19 reference sequence and were obtained from GenBank (http://www.ncbi.nlm.nih.gov). These results were exported from GenomeStudio using the PLINK Input Report Plug-in v2.1.3 by forward strand [31].

For each of the polymorphisms detected in this study the following parameters were assigned: dbSNP IDs (rs numbers), nucleotide position within or relative to the coding sequence based on the NM_000182.4, and amino acid position in the protein for SNPs in the coding sequence based on the reference sequence NP_000173.2. These data were obtained from GenBank (http://www.ncbi.nlm.nih.gov) and were used in this paper as the nomenclature of variants.

#### Variant detections

Among 30 analyzed SNPs we have detected genetic variation for only four variants of *HADHA* gene: rs137852769 (exon 15, missense variant c.1528G>C, p.Glu510Gln), rs7593175 (intron 7, c.573+32T>C), rs146406360 (exon 19, missense variant c.2113G>A, p.Val705Ile) and rs71441018 (exon 7, missense variant c.652G>C, p.Val218Leu).

#### Statistical methods

The observed genotype distribution was determined for all the detected polymorphisms by performing the Hardy-Weinberg equilibrium exact test assuming consistency for a P-value higher than 0.05. Differences in observed MAF values were examined with chi-square test for alleles (with Yates' correction if any allele quantity was below 10) and shown as their P-values, assumed significant if <0.05. The prediction of the effect of aminoacid and nucleotide substitution on protein function or gene were evaluated with the PredictSNP tool [32].

## Results

### Variant c.1528G>C (p.Glu510Gln) of *HADHA* gene (rs137852769)

#### Microarrays method analysis for c.1528G>C—POPULOUS collection (this study)

Out of 5,877 analyzed subjects, 36 (0.61%) were carriers of variants of the *HADHA* gene. We did not find individuals with abnormal homozygous CC genotype and 5,841 (99.39%) were homozygous for the GG genotype. The carriers ratio of this variant in the studied population of Poland was 1/163. After exclusion of individuals from the Pomeranian region the ratio was 1/171. The carriers frequency in the Pomeranian province was 1/103 (Table 1).

**Table 1:** Frequency of *HADHA* c.1528G>C variant carriers observed in this study and combining together with previously published data for Polish population [23].

Voivodeship	number of genotypes—data obtained in this study					number of genotypes—sum of data from this study and data from Piekutowska-Abramczuk et al., 2010***				
	n	GG	GC	CC	ratio GC/n	n	GG	GC	CC	ratio GC/n
Lower Silesian	321*	318	3	0	1:107	574	570	4	0	1:144
Kuyavian-Pomeraian	331*	331	0	0	NA	669	667	2	0	1:335
Lublin	441*	440	1	0	1:441	655	653	2	0	1:328
Lubusz	234*	230	4	0	1:59	440	435	5	0	1:88
Lodz	248*	248	0	0	NA	484	482	2	0	1:242
Lesser Poland	306*	303	3	0	1:102	596	592	4	0	1:149
Masovian	540*	538	2	0	1:270	832	828	4	0	1:208
Opole	227*	227	0	0	NA	404	404	0	0	NA
Subcarpatian	411*	409	2	0	1:206	791	787	4	0	1:198
Podlaskie	233*	231	2	0	1:117	469	465	4	0	1:117
Silesian	965*	960	5	0	1:193	1175	1170	5	0	1:235
Holy Cross (Swietokrzyskie)	81*	80	1	0	1:81	285	284	1	0	1:285
Warmian-Masurian	284*	283	1	0	1:284	616	614	2	0	1:308
Greater Poland	573*	567	6	0	1:96	867	859	8	0	1:108
West Pomeranian	269*	267	2	0	1:135	477	474	3	0	1:159
Pomeranian	413*	409	4	0	1:103	3389	3344	45	0	1:75
All regions of Poland without Pomeranian	5464*	5432	32	0	1:171	9334	9284	50	0	1:187
All regions of Poland with Pomeranian	5877*	5841	36	0	1:163	12723	12705	95	0	1:134
Kashubian population only**	1023	1005	18	0	1:57	1023	1005	18	0	1:57
All data from Pomeranian region with Kashubians	1436	1424	22	0	1:65	4412	4349	63	0	1:70
All regions of Poland with Kashubians	6900	6846	54	0	1:128	13 746	13 633	113	0	1:122

*—data obtained in this study using microarray method,

**—data obtained in this study using pyrosequencing method,

***- TaqMan 5′-nuclease allelic discrimination assay, SSCP analysis

#### Pyrosequencing method analysis for c.1528G>C—Kashubian population (this study)

Out of 1,023 analyzed subjects, 18 (1.75%) were carriers of variants of the *HADHA* gene. We have not found individuals with abnormal homozygous CC genotype and 1,005 (98.25%) were homozygous for the GG genotype. The carriers ratio of this variant in the Kashubian population of Poland was 1/57 (Table 1).

#### Combined data from this study and Piekutowska-Abramczuk et al. (23) for c.1528G>C variant

Out of 9,334 analyzed subjects from all regions, excluding Pomeranians and defined Kashubians, 50 (0.53%) were carriers of variants of the *HADHA* gene. There were no individuals with abnormal homozygous GG genotype and 9,284 (99.47%) were homozygous—GG genotype. The carriers ratio of this variant in the studied population of Poland was 1/187. In the individuals from the Pomeranian region the ratio was 1/75 (without well-defined Kashubians) (Table 1, Fig 3).

**Fig 3:** The frequency of *HADHA* c.1528G>C variant carriers in different regions of Poland.

#### Comparison of c.1528G>C variant frequency in the different Polish regions

Based on pairwise chi-square test for alleles (with Yates correction if any group <10), any significant differences in c.1528G>C variant frequency between particular regions of Poland (excluding the Pomeranian region from this comparison) were detected. Thus, we were able to put together populations from all the regions and compare these pooled data to the Pomeranian population.

By using this methodology, we found that population from the Pomeranian region and Kashubian population on its own significantly differ from the rest of the country in terms of frequency of this variant (p value of chi-square test for alleles p<0.0001) (Table 2).

**Table 2:** Pairwise differences in frequency of c.1528G>C (p.Glu510Gln) variant shown as p-values of chi-square test for alleles (with Yates correction if any subgroup was lower than 10) between populations from all the provinces of Poland, Kashubian population, population of Pomeranian province including/excluding Kashubians and overall population of Poland excluding Pomeranian population. Significant differences (p<0.05) were shaded.

Province of Poland/Group of subjects	subjects	allele G	allele C	LS	KP	Lubl	Lubu	L	LP	M	O	S	P	Sil	HC	WM	GP	WP	(Pom incl K)	K	Pom excl K
**Lower Silesian (LS)**	574	1144	4																		
**Kuyavian-Pomeranian (KP)**	669	1336	2	0.550																	
**Lublin (Lubl)**	655	1308	2	0.568	0.632																
**Lubusz (Lubu)**	440	875	5	0.689	0.183	0.193															
**Łódź (L)**	484	966	2	0.841	0.856	0.840	0.376														
**Lesser Poland (LP)**	596	1188	4	0.763	0.582	0.600	0.647	0.877													
**Masovian (M)**	832	1660	4	0.866	0.886	0.906	0.330	0.804	0.908												
**Opole (O)**	404	808	0	0.241	0.712	0.702	0.090	0.560	0.255	0.389											
**Subcarpathian (S)**	791	1578	4	0.922	0.838	0.858	0.371	0.851	0.964	0.778	0.367										
**Podlaskie (P)**	469	934	4	0.945	0.394	0.409	0.924	0.654	0.987	0.650	0.175	0.702									
**Silesian (Sil)**	1175	2345	5	0.698	0.975	0.997	0.207	0.703	0.739	0.876	0.424	0.934	0.491								
**Holy Cross (HC)**	285	569	1	0.880	0.617	0.607	0.472	0.642	0.910	0.818	0.861	0.859	0.719	0.735							
**Warmian-Masurian (WM)**	616	1230	2	0.620	0.676	0.661	0.224	0.793	0.653	0.965	0.673	0.917	0.454	0.941	0.577						
**Greater Poland (GP)**	867	1726	8	0.869	0.236	0.249	0.942	0.474	0.819	0.426	0.120	0.478	0.862	0.266	0.574	0.288					
**West Pomeranian (WP)**	477	951	3	0.806	0.704	0.722	0.639	0.987	0.767	0.968	0.310	0.917	0.982	0.882	0.997	0.774	0.799				
**Overall from all the provinces (excluding Pomeranian)**	9334	18618	50	-	-	-	-	-	-	-	-	-	-	-	-	-	-	-	6.757x 10^−08^	4.355x 10^−06^	4.659x 10^−06^
**Pomeranian including Kashubians (Pom incl K)**	4412	8761	63	0.217	0.026	0.029	0.778	0.102	0.189	0.040	0.029	0.052	0.420	0.009	0.211	0.038	0.310	0.221			
**Kashubians (K)**	1023	2028	18	0.129	0.013	0.015	0.518	0.059	0.110	0.021	0.016	0.028	0.266	0.004	0.141	0.020	0.176	0.135	0.520		
**Pomeranian exclucing Kashubians (Pom excl K)**	3389	6733	45	0.290	0.039	0.042	0.913	0.136	0.256	0.063	0.037	0.081	0.523	0.017	0.253	0.055	0.432	0.286	0.782	0.386	

#### Comparison of c.1528G>C variant frequency between populations from different countries

Frequency of c.1528G>C was described previously for several populations: Finland, Holland, Estonia and Poland, summarized in Table 3. Taking data from these populations into account the observed frequency does not differ significantly between each other (Table 4). However, the population from the Polish Pomeranian region, either taking the Kashubian subset into account to not, differed significantly from other countries’ populations. No difference, on the border of significance threshold, was only detected between the Dutch and Pomeranian population excluding Kashubians. The Kashubian population on its own had a higher observed frequency of examined SNPs and differed significantly from all compared populations (Table 4).

**Table 3:** Frequency of HADHA 1528G>C mutation carriers in this study and comparison of the previously published data in Poland and different European populations.

	Number of carriers/number of examined persons	Carrier frequency	Source of datas
Netherland	3/2047	1/680	[19]
Finland	5/1200	1/240	[18]
Finland	9/1637	1/181	[33]
Western Finland, Botnia region	3/392	1/132	[33]
Eastern Finland, Noth Karelia	2/385	1/193	[33]]
Northern Finland, Oulu region	1/365	1/365	[33]]
Southern Finland, Helsinki region	3/492	1/164	[33]
Estonia	6/1040	1/173	[17]
Poland (whole country)—children	51/6854	1/189	[23]
Poland, children from whole country without Kashubian region	10/3878	1/389	[23]
Poland, children from Pomeranian region	41/2976	1/73	[23]
Poland, adults from whole country	36/5877	1/163	This study
Poland, adults from Pomeranian region	4/413	1/103	This study
Poland, adults from Kashubian population	18/1023	1/57	This study

**Table 4:** Pairwise differences in frequency of c.1528G>C (p.Glu510Gln) variant shown as p-values of chi-square test for alleles (with Yates correction if any subgroup was lower than 10) between populations from several countries based on literature and population of Pomeranian province including/excluding Kashubians, Kashubian population and overall population of Poland excluding Pomeranian population. Significant differences (p<0.05) were shaded.

Group of subjects / Country	Subjects	allele G	allele C	Pomeranian including Kashubians	Kashubians	Pomeranian exclucing Kashubians	Overall from all the provinces (excluding Pomeranian)	Holland [19]	Finland [18]	Finland [33]	Finland common pool [18, 33]
**Pomeranian including Kashubians**	4412	8761	63								
**Kashubians**	1023	2028	18								
**Pomeranian excluding Kashubians**	3389	6733	45								
**Overall from all the provinces (excluding Pomeranian)**	9334	18618	50								
**Holland** [19]	2047	4091	3	<0.001	<0.001	<0.001	0.031				
**Finland** [18]	1200	2395	5	0.007	0.004	0.015	0.745	0.258			
**Finland** [33]	1637	3265	9	0.008	0.005	0.019	0.912	0.065	0.819		
**Finland common pool** [18, 33]	2837	5660	14	<0.001	<0.001	0.001	0.901	0.075	0.941	0.971	
**Estonia** [17]	1040	2074	6	0.041	0.022	0.070	0.959	0.082	0.812	0.862	0.946

### Other studied polymorphisms of the *HADHA* gene—Microarray data

For rs146406360 (c.2113G>A, p.Val705Ile) polymorphism from 5,879 analyzed people (POPULOUS collection) we found 21 (0.41%) persons with heterozygous GA genotype and no one with AA genotype. The frequency of heterozygotes was 1/280. We did not find any differences in the frequency between all compared provinces of Poland.

For rs7593175 (c.572+32T>C) polymorphism from 5,877 analyzed persons, we found 3,097 with CC (52.70%) genotype, 2,338 with TC (39.78%) genotype and 442 (7.52%) with TT genotype. We did not find any differences in the frequency between different regions of Poland.

Interesting data were uncovered for rs71441018 (c.652G>C, p.Val218Leu) polymorphism. From 5,878 analyzed persons, we found 11 (0.19%) individuals with heterozygous GC genotype. The frequency of heterozygotes within the Polish population was 1/534. Nine of all 11 (82%) detected heterozygotes were found in the Silesian region. The frequency for this region was 1/107, statistically higher than in other regions of Poland (1/2933) (Pearson chi square test, p<0.0001).

### *In silico* prediction of SNP and amino acid substitution effects on protein functionality

*In silico* analysis of SNP effect on protein functionality revealed that all exonic variants, such as rs71441018 (c.652G>C, p.Val218Leu), rs137852769 (c.1528G>C, p.Glu510Gln), rs146406360 (c.2113G>A, p.Val705Ile), have deleterious effects (Table 5). All *in silico* prediction tools for amino acid changes classified the p.Glu510Gln variant as deleterious, and the p.Val218Leu variant was assigned as deleterious by most of them. The p.Val705Ile variant was not predicted as harmful substitution for protein functionality (Table 6).

**Table 5:** Prediction of SNP substitution on pathogenicity, analysis performed *in silico* [32]. Variants predicted by different tools as deleterious were shaded.

			Prediction tool					
Annotation	Genomic position NC_000002.11		PredictSNP2	CADD	DANN	FATHMM	FunSeq2	GWAVA
rs71441018	g.26453084C>G	**Exp. accuracy**	87%	84%	72%	79%	61%	-
		**Prediction**	Deleterious	Deleterious	Deleterious	Deleterious	Deleterious	Unknown
rs137852769	g.26418053C>G	**Exp. accuracy**	87%	84%	71%	72%	61%	51%
		**Prediction**	Deleterious	Deleterious	Deleterious	Deleterious	Deleterious	Deleterious
rs146406360	g.26414385C>T	**Exp. accuracy**	87%	53%	70%	67%	61%	50%
		**Prediction**	Deleterious	Deleterious	Deleterious	Deleterious	Deleterious	Unknown

**Table 6:** Prediction of amino acid substitution on protein functionality, analysis performed *in silico* [32]. Variants predicted by different tools as deleterious were shaded.

			Prediction tool						
Annotation	Amino acid substitution		PredictSNP	MAPP	PhD-SNP	PolyPhen-1	PolyPhen-2	SIFT	SNAP
rs71441018	Val218Leu	**Confidence**	51%	-	61%	67%	40%	79%	55%
		**Pathogenicity**	Deleterious	Unknown	Deleterious	Neutral	Deleterious	Deleterious	Neutral
rs137852769	Glu510Gln	**Confidence**	87%	75%	82%	74%	81%	79%	81%
		**Pathogenicity**	Deleterious	Deleterious	Deleterious	Deleterious	Deleterious	Deleterious	Deleterious
rs146406360	Val705Ile	**Confidence**	74%	85%	89%	67%	47%	65%	83%
		**Pathogenicity**	Neutral	Neutral	Neutral	Neutral	Deleterious	Neutral	Neutral

## Discussion

Kashubians are a relatively small population that inhabits the Pomeranian Province in North Poland. Nowadays, 53,000 native speakers of Kashubian live in Pomerania, although roughly half a million people in Poland claim Kashubian or half Kashubian ancestry.

At the 2011 census however, the number of individuals declaring "Kashubian" as their only identity was 16,000, and 228,000 including those who declared Kashubian and Polish ethnicity. In the same census, over 108,000 people declared everyday use of the Kashubian language [34]. Currently, the number of indigenous Kashubians living in this region is estimated at nearly 230,000. Kashubians are considered to be an isolated population since several lines of evidence suggest that they conform to the criteria of such a population: an old settlement, high rates of endogamy with consanguineous marriages between distant relatives, and slow population expansion with negligible immigration, accompanied by the conservation of a strong socio-cultural identity, including a distinct dialect and traditional customs [27].

Some studies, recently conducted in Poland, employed this isolated population, which is particularly attractive from a genetic point of view. For instance, Siemińska et al. showed, that the variant allele A of rs169969968 of the alpha-5 nicotinic receptor subunit gene (CHRNA5), a polymorphism which is strongly associated with nicotine dependence was significantly less frequent in comparison to the HapMap CEU reference population (www.hapmap.org) [26, 27, 35–37]. Other published genetic studies indicated that Kashubian are very old Polish population, with presence of several mutations/genetic variants almost exclusively detected in patients from this region indicating a founder effect [35, 38–43].

Rebala et al studied the frequencies of Y chromosome haplotypes (7 STR) have found that Kashubian are closely related to similar populations from nearby regions (Kociewie, Kurpie), and also related to other Polish populations, but were different from other Slavics (Lusatia, Chech/Slovakia) and German populations (Meklenburgia, Bavaria) Danish, and Got (Sweden) populations [38].

According to a study published in September 2015, by far the most common Y-chromosome DNA haplogroup among the Kashubians who live in Kashubia, is haplogroup R1a, which is carried by 61.8% of Kashubian males. It is followed in frequency by I1 (13.2%), R1b (9.3%), I2 (4.4%) and E1b1b) (3.4%). Altogether these account for over 9/10 of the total Kashubian Y-DNA diversity. A study from January 2010 discovered similar proportions of most haplogroups (R1a—68.8%, I1—12.5%, R1b—7.8%, I2—3.1%, E1b1b—3.1%), but also found Q1a in 3.1% of Kashubians. This study reported no significant differences between Kashubians from Poland and other Poles in terms of Y chromosome polymorphism. When it comes to mitochondrial DNA haplogroups, according to a January 2013 study, the most common major lineages among the Kashubians, each carried by at least 2.5% of their population, include J1 (12.3%), H1 (11.8%), H* (8.9%), T* (5.9%), T2 (5.4%), U5a (5.4%), U5b (5.4%), U4a (3.9%), H10 (3.9%), H11 (3.0%), H4 (3.0%), K (3.0%), V (3.0%), H2a (2.5%) and W (2.5%). Altogether they account for almost 8/10 of the total Kashubian mtDNA diversity [39–41].

In another study, Lipska et al explored the spectrum of *NPHS2* gene mutations causing steroid-resistant nephrotic syndrome in Polish patients and reported that the carriers of the c.1032delT allele were exclusively found in the Pomeranian (Kashubian) region, suggesting a founder effect origin [42]. Studies of Chmara et al. in the population of patients with hypercholesterolaemia suggested that the (c.662A>G variant in the *LDLR* gene is frequent in this population) [23, 38, 42, 43].

In a 2008 study of Polish newborns a carrier frequency of 1/217 was found, whereas it was significantly higher in the Pomeranian region at 1/73. Because the majority of carriers was detected in children living in the Kashubian region, the authors suggested a probable Kashubian origin (the Kashubian origin of children and parents was not confirmed in that study) of the prevalent c.1528G>C variant. The estimated frequency of disease was 1/16,900 whereas in the rest of Poland it was 1/118,336 [23].

Our study confirms the high frequency of carriers (1/70) of the c.1528G>C variant in the *HADHA* gene within the Pomeranian region (Table 1), and was statistically higher than in other region of Poland (Table 2). The highest frequency was observed in individuals of Kashubian origin at 1/57 which was higher them previously described. In comparison to neighboring countries, (Finland and Estonia) this frequency was also higher. It is interesting that in Finland southern regions have higher frequency of this polymorphism than in northern regions (North Karelia, Oulu vs Helsinki and Bothnia)—Tables 3 and 4 [33].

In our study another region of Poland with high frequency of *HADHA* gene variants was the Lubusz province. This result could be explained by the low number of analyzed persons, and must be verified in enlarged population. When we analyzed the data collected as part of our study together with data from Piekutowska-Abramczuk, the frequency of variant in this region was 1/88 i.e. lower than in Kashubians (Table 1). The frequency observed in Kashubians was statistically higher than in all other region of Poland. For the whole of Poland the carrier frequency 1/122 (113/13,746 analyzed persons)—Table 1.

For other analyzed polymorphism of the *HADHA* gene, prevalence of rs71441018 in the Silesian population was higher compared to the rest of Poland, which had not previously been described. This finding is all the more interesting because this amino acid substitution was classified as deleterious by *in silico* tools and could be clinically significant. More studies are necessary to confirm this observation and explain possible effects on protein functionality.

*In silico* analysis of other polymorphisms showed that predictions for the c.1528G>C (p.Glu510Gln) variant consistent with its previously described clinical significance. Although the effect of the SNP variant c.2113G>A (p.Val705Ile) was also classified as deleterious, amino acid substitution which is vital for protein functionality, was not predicted as negative effect.

## Conclusions

In the summary, the results of our study confirm higher frequency of c.1528G>C variant in *HADHA* gene in the Pomeranian region of North Poland region with the highest frequency in individuals of Kashubian origin, which could confirm founder effect in this population. For the first time we have found a high frequency of rs71441018 polymorphism in the *HADHA* gene within the Silesian population of Southern Poland.
